RETRACTED

# Boswellic Acid Suppresses Growth and Metastasis of Human Pancreatic Tumors in an Orthotopic Nude Mouse Model through Modulation of Multiple Targets

**DOI:** 10.1371/journal.pone.0026943

**Published:** 2011-10-31

**Authors:** Byoungduck Park, Sahdeo Prasad, Vivek Yadav, Bokyung Sung, Bharat B. Aggarwal

**Affiliations:** Cytokine Research Laboratory, Department of Experimental Therapeutics, The University of Texas MD Anderson Cancer Center, Houston, Texas, United States of America; Baylor University Medical Center, United States of America

## Abstract

Pancreatic cancer (PaCa) is one of the most lethal cancers, with an estimated 5-year survival of <5% even when patients are given the best treatment available. In addition, these treatments are often toxic and expensive, thus new agents which are safe, affordable and effective are urgently needed. We describe here the results of our study with acetyl-11-keto-β-boswellic acid (AKBA), an agent obtained from an Ayurvedic medicine, gum resin of *Boswellia serrata.* Whether AKBA has an activity against human PaCa, was examined in *in vitro* models and in an orthotopic nude mouse model of PaCa. We found that AKBA inhibited the proliferation of four different PaCa cell lines (AsPC-1, PANC-28, and MIA PaCa-2 with K-Ras and p53 mutations, and BxPC-3 with wild-type K-Ras and p53 mutation). These effects correlated with an inhibition of constitutively active NF-κB and suppression of NF-κB regulating gene expression. AKBA also induced apoptosis, and sensitized the cells to apoptotic effects of gemcitabine. In the orthotopic nude mouse model of PaCa, p.o. administration of AKBA alone (100 mg/kg) significantly inhibited the tumor growth; this activity was enhanced by gemcitabine. In addition, AKBA inhibited the metastasis of the PaCa to spleen, liver, and lungs. This correlated with decreases in Ki-67, a biomarker of proliferation, and CD31, a biomarker of microvessel density, in the tumor tissue. AKBA produced significant decreases in the expression of NF-κB regulating genes in the tissues. Immunohistochemical analysis also showed AKBA downregulated the expression of COX-2, MMP-9, CXCR4, and VEGF in the tissues. Overall these results demonstrate that AKBA can suppress the growth and metastasis of human pancreatic tumors in an orthotopic nude mouse model that correlates with modulation of multiple targets.

## Introduction

The National Cancer Institute estimated that 18,770 men and 18,030 women in the United States would die of pancreatic cancer (PaCa) in 2010 [1]. Because of a lack of early detection methods and an absence of effective biomarkers, patients with PaCa are usually diagnosed at a late stage, by which time the 5-year survival rate is less than 5% [2]. This low survival rate emphasizes the increased need for effective chemopreventive strategies, early detection methods, and novel treatments. Only 12% of the patients have partial or complete responses to gemcitabine, the standard treatment for advanced PaCa [3], and this treatment is associated with multiple adverse events and drug resistance. Erlotinib, also approved by the U.S. Food and Drug Administration (FDA) to treat pancreatic cancer, does not show significant efficacy either. Thus novel agents that are safe, inexpensive and effective are needed for the treatment of this disease.

RETRACTED

One potential source of novel agents is the large pharmacopeia of traditional medicines. One with promise in the treatment of PaCa is the AKBA (acetyl-11-keto-β-boswellic acid), obtained from the medicinal plant *Boswellia serrata*. It contains beta boswellic acid, a pentacyclic triterpene and the active component of the gum resin (also called frankincense in European pharmacopeia) secreted by the bark of the tree *Boswellia serrata* (Sallai guggul) [4].

AKBA has been used for centuries in traditional Ayurvedic medicine for a wide variety of inflammatory diseases, including inflammatory bowel disease [5] and rheumatoid arthritis [6]. AKBA has been shown to inhibit the growth of a wide variety of tumor cells including glioma [7], colon cancer [8], [9], [10], leukemia cells [11], [12], [13], [14], [15], human melanoma [16], hepatoma [8], and prostate cancer cells [17]. It has been also reported that AKBA has apoptotic effects through a wide variety of mechanisms. AKBA inhibits topoisomerase I and II without inhibiting DNA fragmentation [7], [13], and induces death receptor (DR)-5 but not DR-4 or Fas through increased expression levels of CAAT/enhancer binding protein homologous protein (CHOP), which led to the activation of caspase-8 in prostate cancer cells [18]. The anti-inflammatory effects of this agent were further demonstrated by studies that showed that LPS-induced TNF production is blocked by this drug [19]. Anti-proliferative and anti-inflammatory effects of AKBA are also mediated through the suppression of the NF-κB pathway [20] and STAT3 pathway [21]. More recently our laboratory showed that AKBA can downregulate the expression of CXCR4, a chemokine receptor that has been closely linked with invasion of various cancers [22]. All these studies suggest an anti-inflammatory and anticancer potential for AKBA.

Because several of these targets play a critical role in growth and metastasis of PaCa, we decided to measure the effects of AKBA on a panel of PaCa cell lines and determine whether AKBA alone or in combination with gemcitabine, the current standard of care, affects the growth and metastasis of human pancreatic tumors in nude mice. We found that AKBA inhibited the proliferation and enhanced the apoptosis of gemcitabine in four PaCa cell lines. Moreover, it suppressed the growth and metastasis of human pancreatic tumors in an orthotopic nude mouse model through modulation of multiple targets.

RETRACTED

## Results

### AKBA inhibits the proliferation of pancreatic cancer cells in vitro

We first examined whether AKBA could inhibit the proliferation of human PaCa cell lines. We treated these cell lines with different doses of AKBA for various time periods and determined the inhibition of proliferation by examining mitochondrial activity using the MTT uptake method. As Fig. 1A shows, AKBA suppressed the proliferation of all four pancreatic cancer cell lines in a dose- and time-dependent manner**.** BxPC-3 was most sensitive as 25 µmol/L inhibited proliferation, whereas for the other cell lines, a 50 µmol/L dose was required to fully suppress proliferation.

**Figure 1:** AKBA inhibits proliferation of PaCa cells and enhances the apoptosis of gemcitabine*in vitro*. A, MTT assay results showed dose-dependent suppression of cell proliferation in all four pancreatic cancer cell lines tested. Data are representative of three independent experiments. B, PANC-28 (1×10^6^) cells were treated with AKBA (10, 25, and 50 µmol/L) for 12 h; nuclear extracts were prepared and then assayed for NF-κB activation by EMSA. C, Western blot analysis showed that AKBA inhibited constitutive expression of NF-κB–regulated gene products that regulate antiapoptosis, proliferation, and metastasis in pancreatic cancer cells. The MIA PaCa-2 (1×10^6^) cells were treated with AKBA (10, 25 and 50 µmol/L) for 24 h. Whole-cell lysates were prepared and assayed for NF-κB–regulated gene products by Western blotting. Data represent two independent experiments. D, AKBA potentiates the apoptotic effects of gemcitabine in pancreatic cancer cells *in vitro*. LIVE/DEAD assay results indicated that AKBA potentiates gemcitabine-induced cytotoxicity. Percentages are proportions of apoptotic pancreatic cancer cells. Data are representative of two independent experiments. E, The MIA PaCa-2 (1×10^6^) cells were treated with AKBA (25 µmol/L) for 12 h and then gemcitabine (500 nmol/L) was added for 24 h. Whole-cell lysates were prepared and subjected to Western blotting. Data represent two independent experiments.

### AKBA inhibits constitutive NF-κB activation and NF-κB-regulated proteins in pancreatic cancer cells

We next determined how AKBA inhibits proliferation. Because NF-κB has been linked with proliferation, we examined AKBA's ability to inhibit constitutive NF-κB activation in PANC-28 cell lines. Our results showed that AKBA inhibited constitutive NF-κB activation in PANC-28 (Fig. 1B). We next examined whether AKBA modulates the NF-κB-regulated gene products linked to survival, proliferation, invasion, and angiogenesis. As shown in Figure 1C, AKBA downregulated the expression of antiapoptotic (Bcl-2, Bcl-xL, and survivin), proliferative (COX-2, c-myc, and cyclin D1), and metastatic (MMP-9, CXCR4) proteins in a dose-dependent manner.

RETRACTED

### AKBA potentiates the apoptotic activity of gemcitabine in pancreatic cancer cells

To determine whether AKBA could enhance the apoptotic effects of gemcitabine in these cell lines, we performed the LIVE/DEAD assay, which measures esterase activity. At a dose at which AKBA (25 µmol/L) and gemcitabine (500 nmol/L) alone had minimally apoptotic effects, the two together were highly effective in inducing apoptosis (Fig. 1D). Again BxPC-3 was found to be most sensitive to the combination and MiaPaCa-2 was found to be least sensitive. AKBA also potentiated caspase-mediated cleavage of PARP induced by gemcitabine (Fig. 1E).

### AKBA inhibits the growth of human pancreatic tumors in an orthotopic nude mice model

On basis of our *in vitro* results, we designed studies to determine the effects of AKBA alone and in combination with gemcitabine in human pancreatic tumors orthotopically implanted in nude mice (Fig. 2A). Luciferase-transfected PANC-28 cells were implanted in the tails of the pancreas in nude mice. On the basis of IVIS imaging, the mice were randomized into four groups 1 week later. The treatment was started 1 week after tumor cell implantation and continued per experimental protocol for 4 weeks. The animals were euthanized 6 weeks after tumor cell injection and 5 weeks from the start of treatment. The bioluminescence imaging results indicated a gradual increase in tumor volume in the control group as compared with the three treatment groups (Fig. 2B). The tumor volume in AKBA group was decreased and combination group was significantly lower than in the group treated with AKBA or gemcitabine alone as well as in the vehicle-treated control group (P<0.01). On the 35th day, we euthanized the mice and measured the tumor volume with Vernier calipers. The results were in concordance with those from bioluminescence imaging and showed that the combination reduced the tumor volume more than AKBA did (P<0.01; Fig. 2C and D).

**Figure 2:** AKBA potentiates the effect of gemcitabine in blocking the growth of pancreatic cancer in nude mice. A, schematic of experimental protocol described in *Materials and Methods.* Group I was given corn oil (100 µL, p.o., daily), group II was given AKBA (100 mg/kg, p.o., daily), group III was given gemcitabine (25 mg/kg, i.p., twice weekly), and group IV was given AKBA (100 mg/kg, p.o., daily) and gemcitabine (25 mg/kg, i.p., twice weekly; n = 5). B, bioluminescence IVIS images of orthotopically implanted pancreatic tumors in live, anesthetized mice and measurements of photons per second depicting tumor volume at various time points using live IVIS imaging at the indicated times (n = 5). Points, mean; bars, SEM. C, Necropsy photographs of mice. D, tumor volumes in mice measured on the last day of the experiment at autopsy with Vernier calipers and calculated using the formula V = 2/3πr^3^ (n = 5). Columns, mean; bars, SE.

RETRACTED

### AKBA suppresses distant organ metastasis in mice

We evaluated whether AKBA alone or in combination with gemcitabine can suppress distant organ metastasis in mice. After sacrificing the mice, we found PaCa in the spleen, liver and lungs of vehicle-treated mice; AKBA alone suppressed metastasis to those organs. The combination of AKBA and gemcitabine inhibited metastasis significantly more in these mice and in fact completely suppressed metastasis to the lung (Fig. 3).

**Figure 3:** AKBA potentiates gemcitabine to inhibit distant organ metastasis in orthotopic PaCa nude mice. AKBA and gemcitabine combined inhibited metastases to the spleen, liver, and lungs. Mice were killed, and their abdomen was opened surgically, and then the number of metastasis foci in each organ was counted. Columns, mean; bars, SE.

### AKBA inhibits Ki-67 and CD31 expression

The Ki-67-positive index is used as a marker for cell proliferation, and the CD31 index is a marker for microvessel density. We found that AKBA and gemcitabine downregulated the expression of these biomarkers. AKBA and gemcitabine alone significantly downregulated the expression of Ki-67 in tumor tissues compared with the control group (P<0.05 versus control), and the combination of these two was significantly more effective (Fig. 4A and B). The results also showed that combination of AKBA and gemcitabine remarkably suppressed the expression of CD31 when compared with the control (Fig. 4C and D).

**Figure 4:** AKBA enhances the effect of gemcitabine to inhibit tumor cell proliferation and angiogenesis in PaCa. A, the results of an immunohistochemical analysis of proliferation marker Ki-67 indicated that PaCa cell proliferation was inhibited in mice treated with AKBA alone and in combination with gemcitabine. B, quantification of Ki-67 positive cells was described in *Materials and Methods*. Columns, mean; bars, SE. C, the results of an immunohistochemical analysis of CD31 for microvessel density in PaCa indicated that angiogenesis was inhibited by AKBA alone and in combination with gemcitabine. D, quantification of CD31 positive cells was described in *Materials and Methods*. Columns, mean; bars, SE.

RETRACTED

### AKBA inhibits constitutive NF-κB activation and NF-κB–regulated biomarkers in pancreatic tumors

We next investigated whether the effects of AKBA on tumor growth in mice were associated with the inhibition of NF-κB activation. Fig. 5A shows that AKBA alone suppressed the constitutive activation of NF-κB in the pancreatic tumor tissue, and this down-modulation was enhanced in tissue obtained from animals treated with both AKBA and gemcitabine together.

We also examined expression of various biomarkers in the tumor tissue by western blot. As shown in Fig. 5B, AKBA significantly downregulated the expression of proteins related to antiapoptosis (Bcl-xL), proliferation (cyclin D1, c-myc), metastasis (CXCR4) and invasion (MMP-9, ICAM-1). Especially, expression of Bcl-xL and MMP-9 was reduced more by the combination than just by AKBA.

**Figure 5:** AKBA enhances the effect of gemcitabine against the expression of NF-κB and NF-κB–regulated gene products in pancreatic cancer tissues. A, detection of NF-κB by DNA binding in orthotopic tumor tissue samples showed the inhibition of NF-κB by AKBA. B, Western blot analysis showed that AKBA alone or combination with gemcitabine inhibited the expression of NF-κB–dependent genes. C, immunohistochemical analysis of NF-κB–regulated genes (COX-2, MMP-9, CXCR4 and VEGF) in pancreatic tumor tissues from mice. Percentages indicate positive staining for the given biomarker. Samples from three animals in each group were analyzed, and representative data are shown.

Our immunohistochemical analysis also showed that COX-2, MMP-9, CXCR4 and VEGF expression was downregulated by AKBA, and the combination was even more effective (Fig. 5C).

### AKBA can be detected in plasma and pancreatic tumor tissue

To determine whether AKBA is directly detectable in plasma and pancreatic tissue, serum and PaCa tissue levels of AKBA were examined by HPLC. Serum levels of AKBA were determined 4 h after oral administration of drug in mice. 454±23 ng/ml of AKBA was found in plasma and 273±13 ng/ml of AKBA was found in pancreatic tissue respectively (Fig. 6). These results indicate that there is a strong correlation between tumor regression and the amount of AKBA in the blood.

**Figure 6:** HPLC chromatogram of AKBA in plasma (left) and PaCa tissue (right) in mice.

## Discussion

In the present study, we investigated whether AKBA, a derivative of boswellic acid, could enhance the antitumor activity of gemcitabine against human PaCa. We found that AKBA was highly effective in suppressing the proliferation of various pancreatic cancer cell lines, and when it was combined with gemcitabine, this activity was further enhanced. This activity *in vitro* correlated with the suppression of constitutive NF-κB activation and downregulation of cell survival, proliferative, and metastatic proteins. When examined in an orthotopic model, again AKBA was highly effective in suppressing tumor growth. It was also quite effective in suppressing PaCa metastasis, again in correlation with the downregulation of various biomarkers. The effects of AKBA were more pronounced when it was combined with gemcitabine.

RETRACTED

Ours is the first report to suggest that AKBA can suppress the proliferation and enhance the apoptotic effect of gemcitabine in PaCa cell lines. Gemcitabine alone had a minimal effect on apoptosis in these cell lines. While BxPC-3 cells have been shown to be unaffected by gemcitabine [23], we found that they were highly sensitive to AKBA. This difference may be because BxPC-3 harbors wild-type K-Ras, unlike the other cell lines, in which K-Ras is mutated. The mechanism by which AKBA potentiates the apoptotic effects of gemcitabine may involve suppression of NF-κB. Because NF-κB has been linked with chemoresistance [24], it is very likely that downregulation of NF-κB by AKBA sensitized the cells to gemcitabine. These results agree with a previous report in which MG132, sulfasalazine, and the IκBα super-repressor sensitized pancreatic cancer cells to gemcitabine [23]. NF-kB silencing has been shown to induce apoptosis and increase sensitivity to gemcitabine in a subset of pancreatic cancer cells [25]. Similarly genistein has been shown to sensitize prostate cancer cells to gemcitabine through the downregulation of NF-κB [26].

In addition to these *in vitro* results, we found that AKBA potentiated the antitumor effects of gemcitabine in an orthotopic model of PaCa. Tumor growth was inhibited by almost 50% by 100 mg/kg AKBA alone, and when given in combination with gemcitabine its inhibitory effects were even greater. How AKBA exhibited its effects *in vivo* was investigated in several ways. First, AKBA alone suppressed metastasis of PaCa to the spleen, liver, and lungs. Further, the combination of AKBA and gemcitabine inhibited metastasis significantly in these mice. Second, markers of proliferation (Ki-67) and microvessel density (CD31) were significantly decreased by AKBA. Third, analysis of NF-κB in pancreatic tumors showed that AKBA alone and in combination with gemcitabine inhibited constitutive activation of NF-κB. Fourth, immunohistochemical analysis also showed that AKBA downregulated the expression of proinflammatory biomarker COX-2, suppressed the expression of invasion biomarker MMP-9 and CXCR4, and inhibited the angiogenic biomarker VEGF in the PaCa tissues. All of these effects were further enhanced by gemcitabine. The synergistic effects of the two agents were confirmed by Western blot analysis. Finally, the important aspect of an agent's ability to suppress tumor is the bioavailability, which serves primarily a protective regulatory function constraining diffusion across capillaries in relation to lipid solubility and molecular weight.

RETRACTED

For a successful chemotherapy, agent must be able to reach the blood. AKBA shows high lipid solubility, and we detected it in concentration of 273 ng/ml in PaCa tissues, which corresponded to concentration of 454 ng/ml in the plasma. Thus, these data demonstrate substantial levels of AKBA in PaCa tissue after oral administration and confirm the bioavailability of AKBA. These results are further correlated with the tumor volume regression and decrease in metastases to the spleen, liver, and lungs.

All these potential mechanisms of AKBA we examined, such as inhibition of proliferation, inflammation and metastasis, are related to NF-κB suppression. As we discussed above, because NF-κB has been linked with chemoresistance we would suggest that chemosensitization of PaCa to gemcitabine by AKBA is through an inhibitory effect on NF-κB. Our results are consistent with a recent report in which small hairpin RNA and pharmacological inhibitor of TGF-β-activated kinase (TAK)-1 that activates NF-κB was used to sensitize pancreatic cancer to gemcitabine [27]. Furthermore, it has been reported that NF-κB targeting agent such as curcumin strongly enhanced the antitumor efficacy of radiation [28]. So we propose that AKBA may also sensitize the tumors to radiation therapy.

AKBA has also been shown to bind and inhibit 5-LOX, elastase, and topoisomerase II. AKBA directly inhibits 5-LOX with an IC_50_ as low as 1.5 µM [29]. Further studies have revealed that the pentacyclic triterpene ring structure, hydrophilic group on C4 ring A, and 11-keto functions are all essential for 5-LOX inhibitory activity [30]. Unlike other pentacyclic triterpenes, AKBA has also been shown to inhibit leukocyte elastase with an IC_50_ of 15 µM [31]. Besides 5-LOX and elastase, AKBA was also found to bind to and inhibit topoisomerase (topo) I and II α [32]. The affinity constant (KD) of AKBA for topo I and II α were 70.6 nM and 7.6 nM, respectively. When compared with camptothecin, amascrine or etoposide, AKBA was found to be more potent. Although, we did not measure these proinflammatory and apoptotic biomarkers, it is possible that these also play an important role in the action of AKBA against PaCa.

RETRACTED

Our finding that AKBA downregulated COX-2 expression in pancreatic cancer tissue is notable, as COX-2 is overexpressed in chronic pancreatitis [33] and in human pancreatic cancer tissue. COX-2 expression has been associated with a lower apoptotic index [34], increased cell proliferation [35], increased risk of metastasis [36], [37], and enhanced VEGF production, leading to angiogenesis in pancreatic tumors [38], [39]. Thus inhibition of COX-2 expression in the nude mouse implies that anti-inflammatory effect of AKBA contributes to its anti-tumor effects.

Overall, our results show for the first time that AKBA potentiates the antitumor activity of gemcitabine by modulating multiple biomarkers, leading to the inhibition of proliferation, angiogenesis, invasion, and metastasis. Several clinical trials have been done with AKBA indicating that it is safe agent to use in humans [40], [41]. Our work presented here further provides the basis for clinical trial in patients with pancreatic cancer, one of the most lethal cancers known to mankind.

### Ethics Statement

Our experimental protocol was reviewed and approved by the International Animal Care and Use Committee at University of Texas MD Anderson Cancer Center. Our IACUC protocol number for pancreatic cancer is 10–05–11032.

## Materials and Methods

### Materials

Purified AKBA was supplied by Sabinsa Corp. A 50 mmol/L stock solution of AKBA was prepared and then stored at −20°C as small aliquots until needed. Polyclonal antibodies against cyclin D1, matrix metalloproteinase 9 (MMP-9), survivin, COX-2, c-Myc, Bcl-2, and Bcl-xL were obtained from Santa Cruz Biotechnology. A rabbit polyclonal antibody to CXCR4 was obtained from Abcam. Anti-XIAP antibody was obtained from BD Biosciences. Antiobodies against VEGF and Ki-67 were purchased from Thermo Fisher Scientific. The liquid DAB+ substrate chromogen system–horseradish peroxidase used for immunocytochemistry was obtained from Dako. Penicillin, streptomycin, RPMI 1640, and fetal bovine serum (FBS) were obtained from Invitrogen. Tris, glycine, NaCl, sodium dodecyl sulfate, and bovine serum albumin (BSA) were obtained from Sigma Chemical. Gemcitabine (Gemzar; kindly supplied by Eli Lilly) was stored at 4°C and dissolved in sterile PBS on the day of use.

### Cell lines

The pancreatic cancer cell lines AsPC-1, BxPC-3, MIA PaCa-2, and PANC-28 were obtained from American Type Culture Collection. AsPC-1, PANC-28, BxPC3, and MIA PaCa-2 exhibit K-Ras and p53 mutations, but BxPC-3 harbors wild-type K-Ras. AsPC-1 and BxPC-3 cells were cultured in RPMI 1640 supplemented with 10% FBS, 100 units/mL penicillin, and 100 µg/mL streptomycin. MIA PaCa-2 was cultured in DMEM supplemented with 12% FBS, and PANC-28 was cultured in DMEM supplemented with 10% FBS, 100 units/mL penicillin, and 100 µg/mL streptomycin.

RETRACTED

### Proliferation assay

The effect of AKBA on cell proliferation was determined by the MTT uptake method as follows. The cells (2,000 per well) were incubated with AKBA in triplicate in a 96-well plate and then incubated for 2, 4, or 6 days at 37°C. An MTT solution was added to each well and incubated for 2 hours at 37°C. An extraction buffer (20% SDS and 50% dimethylformamide) was added, and the cells were incubated overnight at 37°C. The absorbance of the cell suspension was measured at 570 nm with an MRX Revelation 96-well multiscanner (Dynex Technologies).

### Apoptosis assay

To determine whether AKBA potentiates the apoptotic effects alone or in combination with gemcitabine in PaCa cells, we used a LIVE/DEAD cell viability assay kit (Invitrogen), which measures intracellular esterase activity and plasma membrane integrity. This assay uses calcein, a polyanionic, green fluorescent dye that is retained within live cells, and a red fluorescent ethidium homodimer dye that can enter cells through damaged membranes and bind to nucleic acids but is excluded by the intact plasma membranes of live cells [42]. Briefly, cells (5,000 per well) were incubated in chamber slides, pretreated with AKBA for 12 hours, and treated with gemcitabine for 24 hours. Cells were then stained with the assay reagents for 30 minutes at room temperature. Cell viability was determined under a fluorescence microscope by counting live (green) and dead (red) cells.

### Animals

Male athymic *nu/nu* mice (4 weeks old) were obtained from the breeding colony of the Department of Experimental Radiation Oncology at University of Texas MD Anderson Cancer Center. The animals were housed in standard Plexiglass cages (five per cage) in a room maintained at constant temperature and humidity and in a 12-hour light/12-hour dark cycle. Their diet consisted of regular autoclave chow and water ad libitum. None of the mice had any lesions, and all were tested pathogen free. Before initiating the experiment, we acclimatized all of the mice to a pulverized diet for 3 days. Our experimental protocol was reviewed and approved by the Institutional Animal Care and Use Committee at University of Texas MD Anderson Cancer Center.

### Orthotopic implantation of pancreatic tumor cells

PANC-28 cells were stably transfected with luciferase as previously described [43]. Luciferase-transfected PANC-28 cells were harvested from subconfluent cultures after a brief exposure to 0.25% trypsin and 0.2% EDTA. Trypsinization was stopped with medium containing 10% FBS. The cells were washed once in serum-free medium and resuspended in PBS. Only suspensions consisting of single cells, with >90% viability, were used for the injections. After mice were anesthetized with ketamine-xylazine solution**,** a small incision was made in the left abdominal flank, and PANC-28 cells (1×10^6^) in 100 µL PBS were injected into the subcapsular region of the pancreas with a 27-gauge needle and a calibrated push button–controlled dispensing device (Hamilton Syringe Co.). A cotton swab was held cautiously for 1 minute over the site of injection to prevent leakage. The abdominal wound was closed in one layer with wound clips (Braintree Scientific, Inc.).

RETRACTED

### Experimental protocol

One week after implantation, the mice were randomized into the following treatment groups (n = 5 per group) based on the bioluminescence first measured with an *in vivo* imaging system (IVIS 200, Xenogen Corp.): (a) untreated control (corn oil, 100 µL daily), (b) AKBA (100 mg/kg once daily p.o.), (c) gemcitabine alone (25 mg/kg twice weekly by i.p. injection), and (d) combination (AKBA, 100 mg/kg once daily p.o., and gemcitabine, 25 mg/kg twice weekly by i.p. injection). Tumor volumes were monitored weekly with the bioluminescence IVIS, which includes a cryogenic cooling unit, and a data acquisition computer running Living Image software (Xenogen Corp.). Before imaging, the animals were anesthetized in an acrylic chamber with 2.5% isoflurane/air mixture and injected i.p. with 40 mg/mL d-luciferin potassium salt in PBS at a dose of 150 mg/kg body weight. After 10 minutes of incubation with luciferin, each mouse was placed in a right lateral decubitus position and a digital grayscale animal image was acquired, followed by the acquisition and overlay of a pseudocolor image representing the spatial distribution of detected photons emerging from active luciferase within the animal. Signal intensity was quantified as the sum of all detected photons within the region of interest per second. The mice were subjected to imaging on days 0, 7, 14, 21, and 28 of treatment. Therapy was continued for 4 weeks, and the animals were euthanized 1 week later. Primary tumors in the pancreas were excised, and the final tumor volume was measured as V = 2/3πr^3^, where r is the mean of the three dimensions (length, width, and depth). Half of the tumor tissue was fixed in formalin and embedded in paraffin for immunohistochemistry and routine H&E staining. The other half was snap frozen in liquid nitrogen and stored at −80°C**.** H&E staining confirmed the presence of tumors in each pancreas.

### Preparation of nuclear extract from tumor samples

Pancreatic tumor tissues (75–100 mg/mouse) from mice in the control and treatment groups were minced and incubated on ice for 30 minutes in 0.5 mL of ice-cold buffer A [10 mmol/L HEPES (pH 7.9), 1.5 mmol/L KCl, 10 mmol/L MgCl_2_, 0.5 mmol/L DTT, and 0.5 mmol/L phenylmethylsulfonyl fluoride (PMSF)]. The minced tissue was homogenized using a Dounce homogenizer and centrifuged at 16,000×g at 4°C for 10 minutes. The resulting nuclear pellet was suspended in 0.2 mL of buffer B [20 mmol/L HEPES (pH 7.9), 25% glycerol, 1.5 mmol/L MgCl_2_, 420 mmol/L NaCl, 0.5 mmol/L DTT, 0.2 mmol/L EDTA, 0.5 mmol/L PMSF, and 2 µg/mL leupeptin] and incubated on ice for 2 hours with intermittent mixing. The suspension was then centrifuged at 16,000×g at 4°C for 30 minutes. The supernatant (nuclear extract) was collected and stored at −70°C until used. Protein concentration was measured by the Bradford assay with BSA as the standard.

RETRACTED

### NF-κB activation in pancreatic cancer cells

To assess NF-κB activation, we isolated nuclei from pancreatic cancer cell lines and tumor samples and carried out electrophoretic mobility shift assays (EMSA) essentially as described next. Briefly, nuclear extracts prepared from pancreatic cancer cells (1×10^6^/mL) and tumor samples were incubated with ^32^P-end-labeled 45-mer double-stranded NF-κB oligonucleotide (4 µg of protein with 16 fmol of DNA) from the HIV long terminal repeat (5′-TTGTTACAA**GGGACTTTC**CGCTG**GGGACTTTC**CAGGGGGAGGCGTGG-3′; boldface indicates NF-κB–binding sites) for 15 minutes at 37°C. The resulting DNA-protein complex was separated from free oligonucleotide on 6.6% native polyacrylamide gels. The dried gels were visualized, and radioactive bands were quantitated with PhosphorImager and ImageQuant software (GE Healthcare).

### Immunohistochemistry of COX-2, MMP-9, CXCR4, and VEGF in tumor samples

The expression of COX-2, MMP-9, CXCR4, and VEGF was determined via an immunohistochemical method described previously [44]. Briefly, pancreatic tumor samples were embedded in paraffin and fixed with paraformaldehyde. After being washed in PBS, the slides were blocked with protein block solution (Dako) for 20 minutes and then incubated overnight with rabbit polyclonal anti-human CXCR4 and anti-MMP-9 (1∶100 for each) or mouse monoclonal anti-human VEGF and anti-COX-2 antibodies (1∶50 and 1∶75, respectively). After incubation with the antibodies, the slides were washed and then incubated with biotinylated link universal antiserum followed by horseradish peroxidase-streptavidin detection with the LSAB+ kit (Dako). The slides were rinsed, and color was developed with 3,3′-diaminobenzidine hydrochloride used as a chromogen. Finally, sections were rinsed in distilled water, counterstained with Mayer's hematoxylin, and mounted with DPX mounting medium (Sigma) for evaluation. Pictures were captured with a Photometrics CoolSNAP CF color camera (Nikon) and MetaMorph software version 4.6.5 (Universal Imaging).

RETRACTED

### Ki-67 immunohistochemistry

Formalin-fixed, paraffin-embedded sections (5 µm) were stained with anti-Ki-67 (rabbit monoclonal clone SP6) antibody as described previously [42]. Results were expressed as the percentage of Ki-67 positive ± SEM per 40× magnification. A total of ten 40× fields were examined and stained cells were counted in three tumors from each of the treatment groups.

### CD31 immunohistochemistry

Ethanol-fixed, paraffin-embedded sections (5 µm) were stained with rat anti-mouse CD31 monoclonal antibodies. Areas of highest microvessel density were then examined under high magnification (100×) and counted. Any distinct area of positive staining for CD31 was counted as a single vessel. Results were expressed as the mean number of vessels ± SEM per high power field (100× magnification). Twenty high-power fields were examined and counted for each of three tumors from each treatment group.

### Western blot analysis

Pancreatic tumor tissues (75–100 mg/mouse) from mice in the control and treatment groups were minced and incubated on ice for 30 minutes in 0.5 mL of ice-cold whole-cell lysate buffer (10% NP40, 5 mol/L NaCl, 1 mol/L HEPES, 0.1 mol/L EGTA, 0.5 mol/L EDTA, 0.1 mol/L PMSF, 0.2 mol/L sodium orthovanadate, 1 mol/L NaF, 2 µg/mL aprotinin, and 2 µg/mL leupeptin). The minced tissue was homogenized with a Dounce homogenizer and centrifuged at 16,000×g at 4°C for 10 minutes. The proteins were then fractionated by SDS-PAGE, electrotransferred to nitrocellulose membranes, blotted with each antibody, and detected by enhanced chemiluminescence reagents (GE Healthcare).

### Measurement of serum and tissue levels of AKBA

AKBA was determined by reverse-phase high performance liquid chromatography (HPLC) on a high-pressure chromatograph equipped with an ultraviolet detector and a 2.0×150-mm column (Gemini C18; particle size, 5 µm, 110A0). The column was eluted in an isocratic flow with a component acetonitrile:methanol:acetic acid (1%) ratio of 70∶20∶10 at an eluent flow rate of 0.35 mL/min. The sample volume was 10 µL. The target compounds were detected at 250 nM. The solution components were identified and quantitatively analyzed using the external standard method with linear regression equations, reliability of approximation (R2), and detection thresholds for AKBA by HPLC. The blood samples were taken from animals 4 h after the administration of AKBA or vehicle. The samples were centrifuged for 20 min at 2000 rpm to obtain the blood plasma, treated with acetone (1.5∶1) for deproteination, and centrifuged again for 15 min at 3000 rpm. The supernatant fraction was separated and extracted with chloroform (2∶1). The chloroform extract was separated, the solvent was removed, and the dry residue was dissolved in methanol and analyzed by HPLC.

RETRACTED

### Statistics

*In vitro* experiments were repeated twice, and statistical analysis was performed. The values were initially subjected to one-way ANOVA, which revealed significant differences between groups, and then later compared between groups with an unpaired Student's t test, which revealed significant differences between two sample means. In vivo experiments were done as at least three independent assays. The values were initially subjected to one-way ANOVA and then later compared among groups with an unpaired Student's t test.
